# Puerarin 6″‐O‐xyloside suppressed HCC via regulating proliferation, stemness, and apoptosis with inhibited PI3K/AKT/mTOR

**DOI:** 10.1002/cam4.3285

**Published:** 2020-07-21

**Authors:** Long Li, Jun‐Dong Liu, Guo‐Dong Gao, Kai Zhang, Yu‐Wei Song, Hong‐Bo Li

**Affiliations:** ^1^ Department of General Surgery People's Hospital of Rizhao Rizhao Shandong Province China

**Keywords:** KDM6B, liver cancer, mTOR, PI3K, Puerarin 6″‐O‐xyloside

## Abstract

Puerarin 6″‐O‐xyloside is a tumor suppressive derivate of Puerarin that is recently characterized as a lysine‐specific demethylase 6B inhibitor. Here we investigated the effects of Puerarin 6″‐O‐xyloside in hepatocellular carcinoma (HCC) cell lines SMMC‐7721 and HepG2. Cell viability, proliferation, stemness, protein expression, and autophagy were tested by CCK‐8, colony formation, sphere formation, western blotting, and LC3B GFP puncta per cell, respectively. Apoptosis, CD133‐positive cells, and JC‐1‐labeled mitochondrial membrane potential were measured by flow cytometry. The effects of Puerarin 6″‐O‐xyloside in vivo were explored in HepG2 xenograft mice. Puerarin 6″‐O‐xyloside inhibited cell viability, proliferation, and stemness, and promoted apoptosis in both SMMC‐7721 and HepG2 cells. Further experiments showed promoted autophagy and decreased mitochondrial membrane potential, and decreased expression of p‐PI3K, p‐AKT, and p‐mTOR in HepG2 cells. Co‐administration of 3‐MA with Puerarin 6″‐O‐xyloside obviously augmented these effects including inhibited protein expression of p‐PI3K, p‐AKT, and p‐mTOR, and inhibited proliferation, promoted apoptosis, and decreased stemness. In HepG2 xenograft mice, 100 mg/kg/d Puerarin 6″‐O‐xyloside significantly suppressed tumor growth, stemness, and apoptosis. In conclusion, our study indicated that Puerarin 6″‐O‐xyloside decreased cell viability, proliferation, and stemness, and promoted autophagy and mitochondria‐dependent apoptosis of HCC, at least partly through inhibiting PI3K/AKT/mTOR. These results highlighted Puerarin 6″‐O‐xyloside as a promising prodrug that could inhibit both PI3K/AKT/mTOR and epigenetic demethylation.

## Graphical abstract

Puerarin 6″‐O‐xyloside suppressed HCC via regulating proliferation, stemness, autophagy, and apoptosis with inhibited PI3K/AKT/mTOR pathway. Puerarin 6″‐O‐xyloside targeted PI3K, mTOR, and KDM6B.

## 1 INTRODUCTION

Liver cancer is among the leading causes of cancer deaths worldwide, accounting for 854 000 incidences and 810 000 deaths globally in 2015, and hepatocellular carcinoma (HCC) is the most common subtype.^1^ Early diagnosis is the only hope for liver cancer at present as only limited therapeutic strategies for late‐stage conditions are present.^2^ With the transmission of hepatitis B virus and influence of other risk factors, and burden of liver cancer increased, more effective therapies for diagnosis and treatment of HCC are in urgent need to be developed.

Natural agents derived from plants are important sources of prodrug. Puerarin 6″‐O‐xyloside is a major compound in the root of the famous Traditional Chinese Medicine Pueraria lobata (Willd.) Ohwi (P. lobata).^3^ Puerarin 6″‐O‐xyloside is formed with substitution of hydroxyl group at C‐6″ of Puerarin with a xylose residue (Figure 1A). Puerarin 6″‐O‐xyloside and Puerarin were reported to be tumor suppressive for several carcinomas including esophageal cancer,^4^ gastric carcinoma,^5^ lung carcinoma,^6^ colon cancer, and HCC.^7^, ^8^ In mouse models of xenograft esophageal and gastric tumors, Puerarin exhibited equally potent efficiency with 5FU, and co‐administration of Puerarin and 5FU exhibited even better with no significant adverse effect seen.^4^, ^5^ Researches about Puerarin 6″‐O‐xyloside and Puerarin were not seen in the same cell or animal model. Anyway Puerarin 6″‐O‐xyloside could be more effective as its median inhibitory concentration (IC50) reported is usually about 40 μg/mL while IC50 of Puerarin is about 500 μg/mL.^6^, ^7^ Especially, Puerarin 6″‐O‐xyloside showed obvious safety in mice and rats with a dose of 80 mg/kg each day in vivo.^9^ Puerarin inhibited proliferation and promoted mitochondrial‐mediated apoptosis in SMMC‐7721 cells, mainly through inhibiting MAPK signaling.^7^, ^10^ Similarly, Puerarin 6″‐O‐xyloside was proved to be effective to lung and colon cancers, mainly through induction of apoptosis.^6^, ^8^ Puerarin 6″‐O‐xyloside‐induced apoptosis was characterized by upregulated cleaved caspase‐3, cleaved caspase‐9, B‐cell lymphoma 2 (Bcl‐2)‐associated X protein and phosphorylated c‐Jun terminal kinase, and downregulated Bcl‐2, matrix metalloproteinase (MMP)‐3, and MMP‐9.^6^ These highlighted the involvement of mitochondria in Puerarin 6″‐O‐xyloside‐induced apoptosis.

**FIGURE 1:** Effects of Puerarin 6″‐O‐xyloside on HCC cell lines. A, The structure of Puerarin and Puerarin 6″‐O‐xyloside. Both SMMC‐7721 and HepG2 cells were seeded in 96‐well plates at a density of 3000 cells/well. Increasing concentrations of Puerarin 6″‐O‐xyloside were added after 24 h and incubated for another 24 h before CCK‐8 was added and tested. B, Cell viability of SMMC‐7721 and HepG2 cells treated with Puerarin 6″‐O‐xyloside. *P < .05 compared with no Puerarin 6″‐O‐xyloside treatment analyzed by one‐way ANOVA. Data were from three independent replicates

The mechanism of action of Puerarin 6″‐O‐xyloside is still largely unknown other than induced apoptosis. Compared to Puerarin, antitumor activity of Puerarin 6″‐O‐xyloside largely improved. But Puerarin 6″‐O‐xyloside is far from perfect for it could be easily hydrolyzed. Puerarin has been approved to induce apoptosis in SMMC‐7721 cells; then Puerarin 6″‐O‐xyloside may also be effective to liver cancer cells as Puerarin 6″‐O‐xyloside is a derivate of Puerarin. In this study, we investigated the possible effects of Puerarin 6″‐O‐xyloside on both SMMC‐7721 and HepG2 cells, concerning proliferation, apoptosis, stemness, and autophagy and possibly related signaling pathways.

## 2 RESULTS

### 2.1 Puerarin 6″‐O‐xyloside dose dependently inhibited cell viability in SMMC‐7721 and HepG2 cells

To establish the effects of Puerarin 6″‐O‐xyloside, CCK‐8 was carried out in normal liver cell line LO2 and liver cancer cell lines SMMC‐7721 and HepG2. As shown in Figure 1B, no significant change in viability was seen in LO2 treated with up to 400 μmol/L of Puerarin 6″‐O‐xyloside. 50 and 100 μmol/L of Puerarin 6″‐O‐xyloside started to show significant inhibition of cell viability in HepG2 and SMMC‐7721 cells, respectively. Overall, HepG2 cells were slightly more sensitive to Puerarin 6″‐O‐xyloside treatment. The calculated IC50 of Puerarin 6″‐O‐xyloside in SMMC‐7721 is about 109 μmol/L and IC50 in HepG2 is about 57 μmol/L. To explore the possible mechanism of action of Puerarin 6″‐O‐xyloside in liver cancer, 0, 5, 10, and 20 μmol/L of Puerarin 6″‐O‐xyloside (indicated as POX 0, POX 5, POX‐10, and POX 20 μmol/L in figures) were chosen for their miner toxicity in later experiments.

### 2.2 Puerarin 6″‐O‐xyloside inhibited proliferation and promoted apoptosis in SMMC‐7721 and HepG2 cells

Proliferation and apoptosis are most common downstream of chemicals that harbor antitumor effects. We tested the effect of Puerarin 6″‐O‐xyloside on proliferation and apoptosis of SMMC‐7721 and HepG2 cells. Colony formation assay showed dose‐dependent inhibition of proliferation with Puerarin 6″‐O‐xyloside both in SMMC‐7721 and HepG2 cells as shown in Figure 2A,B, as well as indicated by western blotting of proliferation marker protein Ki67 shown in Figure 2E. Similar to cell viability results, proliferation inhibition in HepG2 cells was more significant than that in SMMC‐7721. Cell apoptosis and cell necrosis were dose dependently induced by Puerarin 6″‐O‐xyloside in both cell lines as shown in Figure 2C,D. Again, apoptosis in HepG2 cells was more significant than in SMMC‐7721, with 5 μmol/L in HepG2 vs 10 μmol/L in SMMC‐7721 started to obviously (*P* < .05 vs 0 μmol/L) induce apoptosis. The increased apoptosis was also validated by the increased ratio of cleaved caspase‐3 to caspase‐3 as shown in Figure 2F.

**FIGURE 2:** Puerarin 6″‐O‐xyloside inhibited proliferation and promoted apoptosis in SMMC‐7721 and HepG2 cells. Both cell lines were treated with 0, 5, 10, and 20 μmol/L of Puerarin 6″‐O‐xyloside for 24 h. The proliferation was shown with crystal violet staining (A) and area of the staining was measured by ImageJ (B). Flow cytometry was applied to show apoptotic cells (C) and the number of apoptotic cells was counted (D). Western blotting was used to show relative protein expression of Ki67 (E) and the ratio of cleaved caspase‐3 to caspase‐3 (F) in both cell lines. *P < .05 and **P < .01 compared with no Puerarin 6″‐O‐xyloside treatment by *t* test of at least three replicates. POX: Puerarin 6″‐O‐xyloside

### 2.3 Puerarin 6″‐O‐xyloside reduced stem‐like property of SMMC‐7721 and HepG2 cells

Stem‐like property of SMMC‐7721 and HepG2 cells treated with Puerarin 6″‐O‐xyloside was estimated by sphere formation, CD133 enabled cell‐sorting, and protein expression of stemness marker OTC4. Puerarin 6″‐O‐xyloside dose dependently reduced the formation of spheres, and decreased the size and number of spheres (Figure 3A‐C). With the dosage increase, the number of CD133‐labeled cells was increased both in HepG2 and SMMC‐7721 cells (Figure 3D,E). The inhibition of stem‐like property of Puerarin 6″‐O‐xyloside in both cell lines was also validated by the dose‐dependent decrease of OCT4 protein (Figure 3F). Stem‐like property in HepG2 cells was more easily inhibited by Puerarin 6″‐O‐xyloside compared to SMMC‐7721, which was similar to trends in proliferation.

**FIGURE 3:** Stem‐like property of SMMC‐7721 and HepG2 cells treated with Puerarin 6″‐O‐xyloside. Both cell lines were treated with 0, 5, 10, and 20 μmol/L of Puerarin 6″‐O‐xyloside for 10 d. (A) Sphere formation assay was used to test the effects of Puerarin 6″‐O‐xyloside treatment to stemness. Diameter (B) and the number of spheres per 100 cells (C) were measured. (D) CD133‐positive cells tested by anti‐CD133‐PE powered flow cytometry. (E) Number of CD133‐positive cells. (F) Relative protein expression of OCT4 tested by western blotting. *P < .05 and **P < .01 compared with no Puerarin 6″‐O‐xyloside treatment by *t* test of at least three replicates. POX: Puerarin 6″‐O‐xyloside

### 2.4 Puerarin 6″‐O‐xyloside induced autophagy and reduced mitochondrial membrane potential in HepG2 cells

Apoptosis is downstream of most anticancer therapeutics. To investigate the induction and modulation of apoptosis by Puerarin 6″‐O‐xyloside, autophagy and mitochondrial membrane potential were tested. Puerarin 6″‐O‐xyloside induced similar effects in HepG2 cells and SMMC‐7721 cells including inhibition of cell viability, proliferation, and sphere formation, with HepG2 cells slightly more sensitive to Puerarin 6″‐O‐xyloside treatment. So in the following experiments, further mechanism of action of Puerarin 6″‐O‐xyloside in liver cancer was assessed in HepG2 cells. As indicated in Figure 4A, Puerarin 6″‐O‐xyloside dose dependently promoted LC3‐positive puncta per cell in HepG2 cells, with significant difference observed at 5 μmol/L group (*P* < .05), and more significant difference seen at 20 μmol/L group (*P* < .01). The promotion of autophagy by Puerarin 6″‐O‐xyloside was also validated by autophagy‐related proteins as shown in Figure 4B. Autophagy was significantly induced with 5‐μmol/L Puerarin 6″‐O‐xyloside (*P* < .05) and very significantly induced at 20 μmol/L (*P* < .01), as indicated by the ratio of LC3BII/LC3BI, and protein expression of Beclin 1 and ATG7.

**FIGURE 4:** Change in autophagy and mitochondrial membrane potential with treatment of Puerarin 6″‐O‐xyloside in HepG2 cells. GFP‐LC3 plasmid was transfected into HepG2 cells, then treated with 0, 5, 10, and 20 μmol/L of Puerarin 6″‐O‐xyloside for 24 h and (A) LC3 puncta per cells were counted with Image Pro Plus, Blue fluorescence form DAPI and green fluorescence were GFP‐LC3B. (B) Relative expression of autophagy‐related proteins in cells tested by western blotting. (C) Mitochondrial membrane potential measured by JC‐1‐labeled flow cytometry. When mitochondrial membrane potential loss happens, JC‐1 in cytoplasm captures the leaked proton and turns green. *P < .05 and **P < .01 compared with no Puerarin 6″‐O‐xyloside treatment by *t* test of at least three replicates. POX: Puerarin 6″‐O‐xyloside

Then Puerarin 6″‐O‐xyloside‐induced decrease of mitochondrial membrane potential was measured by JC‐1‐labeled flow cytometry. The results showed that mitochondrial membrane potential was dose dependently decreased in Puerarin 6″‐O‐xyloside‐treated HepG2 cells, as indicated by increased green fluorescence in Figure 4C.

### 2.5 PI3K/AKT/mTOR is involved in the mechanism of action of Puerarin 6″‐O‐xyloside in HepG2 cells

As stem‐like property was inhibited in both cell lines and autophagy was induced in HepG2 cells with treatment of Puerarin 6″‐O‐xyloside, typical proteins of PI3K/AKT/mTOR, which participate in both stemness and autophagy regulation, were tested (Figure 5A,B). Treatment with Puerarin 6″‐O‐xyloside in HepG2 cells dose dependently inhibited p‐PI3K p85, PI3K p110α, p‐AKT, and p‐mTOR expression, with significant difference observed with 5 μmol/L of Puerarin 6″‐O‐xyloside (*P* < .05). Then, 20 μmol/L of Puerarin 6″‐O‐xyloside and 1‐mM 3‐MA were used to show its effects through inactivated PI3K. PI3K, AKT, and mTOR were all inhibited by Puerarin 6″‐O‐xyloside and 3‐MA, and co‐administration of Puerarin 6″‐O‐xyloside and 3‐MA more significantly inhibited PI3K/AKT/mTOR signaling (Figure 5A,C). Treatment with Puerarin 6″‐O‐xyloside or 3‐MA reduced proliferation of HepG2 cells, and a more significant inhibition was observed when co‐administered (Figure 5D,E). Cell apoptosis was induced by Puerarin 6″‐O‐xyloside or 3‐MA, and more obviously induced by Puerarin 6″‐O‐xyloside and 3‐MA (Figure 5F,G). Similar trend was observed in stem‐like property; both diameter and number of spheres per 100 cells were reduced by Puerarin 6″‐O‐xyloside or 3‐MA, and co‐administration of the two indicated a more significant reduction (Figure 5H‐J). These results showed that the inhibited proliferation, promoted apoptosis, and reduced stemness by Puerarin 6″‐O‐xyloside were enhanced by 3‐MA.

**FIGURE 5:** Effects of 3‐MA to Puerarin 6″‐O‐xyloside‐treated HepG2 cells. A, Relative protein expression of PI3K/AKT/mTOR and their phosphorylated form in HepG2 treated with 0, 5, 10, and 20 μmol/L of Puerarin 6″‐O‐xyloside for 24 h. Then HepG2 cells were treated with PBS (control), Puerarin 6″‐O‐xyloside (POX 20 μmol/L), 1 mmol/L of 3‐MA or Puerarin 6″‐O‐xyloside + 3‐MA (POX 20 μmol/L + 3‐MA) for 24 h. B, Relative PI3K/AKT/mTOR pathway protein expression in HepG2 cells treated with 3‐MA and/or Puerarin 6″‐O‐xyloside. C, and D, Cell proliferation indicated with crystal violet staining. E and F, Apoptosis measured by flow cytometry. Stemness was indicated by sphere formation assay G, and diameter of sphere H, and number of spheres per 100 cells I, were measured. *P < .05 compared with control and ^#^ *P* < .05 compared with Puerarin 6″‐O‐xyloside treatment by *t* test of at least three replicates. POX: Puerarin 6″‐O‐xyloside

### 2.6 Puerarin 6″‐O‐xyloside inhibited tumor progression in HepG2 xenograft mice

To further validate the effects of Puerarin 6″‐O‐xyloside on liver cancer, Balb/c nude mice were used to establish HepG2 xenograft tumors and were treated with 100 mg/kg/d of Puerarin 6″‐O‐xyloside for 28 days. As a result, Puerarin 6″‐O‐xyloside significantly reduced the tumor volume (Figure 6A,B). The expression of Ki67 and OCT4 was reduced in Puerarin 6″‐O‐xyloside‐treated mice, while apoptosis was induced in Puerarin 6″‐O‐xyloside‐treated mice (Figure 6C,D). The results verified that Puerarin 6″‐O‐xyloside inhibited progression of liver cancer in vivo.

**FIGURE 6:** Effects of Puerarin 6″‐O‐xyloside in HepG2 Xenograft Balb/c mice. The mice were treated with saline or 100 mg/kg/d for 28 d. A, The tumors harvested. B, The volumes of the tumors were measured. C, The tumors were stained as indicated to show proliferation, stemness, and apoptosis. D, The staining of Ki67, OCT4, and TUNEL was semi‐quantified

## 3 MATERIALS AND METHODS

### 3.1 Cell culture and reagents

LO2, HepG2, and SMMC‐7721 were obtained from the American Type Culture Collection (ATCC), maintained in DMEM (Invitrogen) supplemented with 10% FBS (Invitrogen) and antibiotics (1% penicillin and 100 μg/mL streptomycin; Beyotime), with an atmosphere containing 5% CO2 at 37°C. JC‐1 (T4069) and 3‐MA (M9281) were from Sigma‐Aldrich, Puerarin 6″‐O‐xyloside was purchased from Tauto Biotech (E‐1160, Shanghai, China), and Cell Counting Kit 8 (CCK‐8, C0037), PBS, Crystal Violet Staining Solution (C0121), 4% Paraformaldehyde Fix Solution, Colorimetric TUNEL Apoptosis Assay Kit and Bicinchoninic acid (BCA) protein assay reagent (P0012S) were purchased from Beyotime. Mouse CD133‐PE antibody was purchased from Miltenyi Biotec; antibodies of Ki67 (ab15580), Cleaved Caspase‐3 (ab32042), Caspase‐3 (ab90437), OCT4 (ab109183), LC3B (ab229327), Beclin1 (ab207612), ATG7 (ab133528), AKT (ab18785), p‐AKT (ab8933), mTOR (ab32028), and p‐mTOR (abs) were purchased from Abcam. PI3K p110α (#4255), PI3K p85 (#4257), p‐PI3K p85 (#4228), GAPDH (#5174) antibodies and all secondary antibodies were purchased from CST (Danvers, MA, USA). Annexin V fluorescein isothiocyanate/propidium iodide (FITC/PI) kit was purchased from BD Biosciences. Other reagents were purchased from Beyotime and Solarbio.

### 3.2 Cell viability assay

LO2, HepG2, and SMMC‐7721 cells were seeded in 96‐well plates at a density of 5 × 10^5^ cells/well in 100‐μL medium. After cultured for 24 hours, cells were changed with another 100‐μL medium containing Puerarin 6″‐O‐xyloside (0, 0.1, 0.2, 0.5, 1, 2, 5, 10, 20, 50, 100, 200, 300, and 400 μmol/L). After incubation for more than 22 hours, 10 μL of CCK‐8 was added to each well. Optical density was measured at 450 nm, 2 hours after CCK‐8 was added. The inhibitory rate was calculated according to the following formula: [(ODC0 − ODCx)/(ODC0 − ODPBS)] × 100%. Outliers were discarded by G test. Four replicate wells were involved in each concentration. The experiment was independently repeated for 3 times.

### 3.3 Colony formation assay

About 1000 cells were seeded in 6‐well plates. After stable adhesion formed, medium containing Puerarin 6″‐O‐xyloside (0, 5, 10, 20 μmol/L, 2 mL) was added and refreshed every 3‐4 days. After incubated for 14 days, each well was washed twice with PBS, fixed with methanol for 30 minutes, and then stained with 0.5% crystal violet for 30 minutes at room temperature. The test was performed in triplicate. Images were acquired using a digital camera.

### 3.4 Sphere formation assay

HepG2 and SMMC‐7721 cells were seeded in low adherent 24‐well culture plates at 2 × 10^3^ cells per well. Then, cells were incubated in serum‐free medium of RPMI 1640 containing 20 μL/mL of B27, 20 ng/mL of EGF, 20 ng/mL of bFGF, and 1% of penicillin‐streptomycin. After incubation at 37°C in a 5% CO2 incubator for 10 days, pictures were taken under a microscope and the number of spheres was counted in three separate 40 × fields.

### 3.5 Flow cytometry

Flow cytometry analysis was applied to show apoptosis, stem‐like property, and change in mitochondrial membrane potential. In brief, HepG2 and/or SMMC‐7721 cells were treated with different dose of Puerarin 6″‐O‐xyloside (0, 5, 10, and 20 μmol/L) for 24 hours before tested. Apoptosis was tested as previously reported. ^11^ Cells were digested with 2.5% trypsin, harvested in flow cytometry tubes, and centrifuged for 5 minutes at 500 g. Cell pellets were incubated with Annexin V‐FITC for 15 minutes and then with PI for 10 minutes, and analyzed with a FACScan flow cytometer (BD Biosciences). Annexin V‐FITC‐positive cells were considered apoptotic cells and PI‐positive cells are considered dead cells.^12^

For analysis of stem‐like property, fluorescence‐activated cell sorting (FACS) assay was performed. For each well, 100 μL of 1 × 10^7^ cells was incubated with 10‐μL anti‐CD133‐PE in the dark at 4°C for 10 minutes. Then, cells were washed twice with buffer and suspended in 500 μL of buffer for analysis by flow cytometry.

For analysis of mitochondrial membrane potential, cells were detached by trypsinization, re‐suspended with JC‐1 working solution, incubated in 37°C, 5% CO2 for 15 minutes, then re‐suspended again in PBS, and analyzed with FACScan as described previously.^13^, ^14^

### 3.6 Western blotting

Cells were lysed under ice in 20 μL of cold RIPA Lysis Buffer. Protein lysis was collected and BCA method was adopted to adjust protein concentrations. About 30 μg of total protein per sample was used in electrophoresis. Primary antibodies were incubated shaken at 4°C overnight, and secondary antibodies were incubated at room temperature for 1 hour. Images were collected using the Gel Imaging System (Bio‐Rad) with ECL and analyzed by ImageJ.

### 3.7 GFP‐LC3 plasmid transfection and confocal microscopy

HepG2 cells underwent GFP‐LC3 plasmid transfection that was performed using Lipofectamine 3000 transfection reagent (Invitrogen, L3000) according to the manufacturer's protocol. GFP‐LC3 plasmids were bought from Addgene (#24920). After incubation for 48 hours, the medium containing the transfection mixture was replaced with fresh complete medium and the cells were treated with Puerarin 6″‐O‐xyloside (0, 5, 10, 20 μmol/L, 2 mL) for 24 hours, then viewed by a laser scanning confocal microscope (Zeiss). Then images were analyzed by ImageJ.

### 3.8 Animal experiments

Male Balb/c mice (6 weeks old, weighing ~20 g) were purchased from and in vivo experiments were applied at Hunan SJA Laboratory Animal Co., Ltd. The mice were housed under a specific‐pathogen‐free (SPF) environment with a 12‐hour light/dark cycle and free access to food and water.

A total of 10 mice were randomly divided into two groups. About 1 × 10^7^ HepG2 cells were subcutaneously injected into the right dorsal area of each mice. The experiment group mice were intraperitoneal injected with 100 mg/kg/d of Puerarin 6″‐O‐xyloside in saline; the control group mice were injected with equivalent saline.^6^, ^9^ After 28 days, the mice were sacrificed and the tumors were harvested. After photographing, the tissues were fixed in 4% Paraformaldehyde Fix Solution. The fixed tissues were paraffin‐embedded to get 5‐μm slides before rehydration. Then the slides were stained with TUNEL, Ki67, and OCT4 antibodies, respectively, according to the manufacturer's instructions and observed with a fluorescence microscope (Olympus) and analyzed with Image Pro Plus (version 6.0, Media Cybernetics).

### 3.9 Statistical analysis

Statistical analyses were performed with GraphPad Prism 6.0. Images were quantified by ImageJ or Image Pro Plus software. Data were analyzed with *t* tests or one‐way analysis of variances (ANOVA). *P* < .05 was taken as statistically significant.

## 4 DISCUSSION

Puerarin 6″‐O‐xyloside has been indicated to be effective to lung and colon cancers.^6^, ^8^ Here we suggested that Puerarin 6″‐O‐xyloside was also effective to HCC in a dose‐dependent manner, as indicated in both SMMC‐7721 and HepG2 cells in vitro, and in HepG2 Xenograft mice. Main effects of Puerarin 6″‐O‐xyloside on HCC cell lines include inhibited proliferation and stemness, and promoted autophagy and apoptosis. Inhibition of cell viability in HCC cells in this study was about 120 μmol/L which seemed to be relatively higher than 40 μmol/L in SW480, LoVo, HCT‐116, and A549 cells. This could be a result of different cell lines, possible drug conditions, and cell culture conditions. Puerarin exhibited no significant liver toxicity in nude mice at 30 mg/kg/day.^5^ Puerarin 6″‐O‐xyloside, in contract, was safe at 60 mg/kg/day for 12 weeks in ICR mice.^9^ This remarkable safety was predictable, as no toxic group was introduced and the hydroxyl‐rich structure could be easy to be eliminated directly. In the current research, 100 mg/kg/day of Puerarin 6″‐O‐xyloside was used in Balb/c mice. As a result, Puerarin 6″‐O‐xyloside showed significant antitumor effects without observable toxicity. These strongly supported the possible application of Puerarin 6″‐O‐xyloside in tumors, especially in HCC.

Antitumor effects of Puerarin 6″‐O‐xyloside could be more than apoptosis. In this study, Puerarin 6″‐O‐xyloside‐inhibited proliferation was indicated by colony formation assay. Apoptosis was induced with Puerarin 6″‐O‐xyloside as indicated by flow cytometry and relative protein expression of cleaved caspase‐3. Stem‐like property was decreased by Puerarin 6″‐O‐xyloside as indicated by sphere formatting assay, number of CD133‐positive cells, and relative protein expression of stemness marker OCT4. All these effects were observed in both SMMC‐7721 and HepG2 cells in a dose‐dependent manner. These results indicated that targets of Puerarin 6″‐O‐xyloside in HCC could be complex.

Autophagy is an important regulator of apoptosis especially in the mechanism of action of antitumor therapeutics. Although autophagy is induced by drugs to initiate apoptotic cell death in vitro, autophagy enables tumor cells to evade damages from drugs in vivo.^15^ Knockout of autophagy‐related gene promoted incidence of premalignant lesions, while prevented established malignant tumors. This phenomenon was also validated in HCC.^16^ Though inhibition of autophagy in late‐stage cancers possibly would impair hematopoiesis and/or systemic immunity, co‐administration of autophagy inhibitory drugs with other therapeutics is currently being pursued for late‐stage cancers.^15^ In the present study, we observed that Puerarin 6″‐O‐xyloside‐induced autophagy in HepG2 cells, and inhibition of autophagy with 3‐MA significantly enhanced inhibition of proliferation and stemness, and promotion of apoptosis. These results highlighted that autophagy was possibly induced to reduce toxicity of Puerarin 6″‐O‐xyloside, and autophagy inhibitors could be a potent adjuvant for Puerarin 6″‐O‐xyloside in HCC treatment.

Mitochondria‐induced apoptosis, the predominant mechanism for targeted chemotherapy, was also indicated to be involved in the mechanism of action of Puerarin 6″‐O‐xyloside in previous studies.^6^ Loss of mitochondrial membrane potential is an early hallmark of mitochondria‐induced apoptosis. Upon loss of mitochondrial membrane potential, proapoptotic molecules in mitochondria, such as cytochrome c, were released out to the cytoplasm. Then, the released proapoptotic molecules interacted with adenosine triphosphate, apoptotic protease activating factor 1, and caspase‐9, and subsequently activated caspase‐3, which consequently elicited caspase‐dependent apoptotic cell death.^17^ In both SMMC‐7721 and HepG2 cells, apoptosis was dose dependently induced with Puerarin 6″‐O‐xyloside. Further experiments showed that loss of mitochondrial membrane potential was induced by Puerarin 6″‐O‐xyloside. These indicated the involvement of mitochondria in Puerarin 6″‐O‐xyloside‐induced apoptosis in HCC.

The in vivo anti‐lung cancer effects of Puerarin 6″‐O‐xyloside were simply characterized previously.^6^ Here, we investigated the effects of Puerarin 6″‐O‐xyloside in HepG2 Xenograft Balb/c nude mice. As currently maximum dosage of Puerarin 6″‐O‐xyloside (80 mg/kg/d) reported no toxicity,^9^ 100 mg/kg/d was employed. Administration of Puerarin 6″‐O‐xyloside significantly reduced tumor volume with 28 days. What is more, expression of KI67 and OCT4 was inhibited and apoptosis was induced in tumors of the treated mice. The in vivo experiments supported that Puerarin 6″‐O‐xyloside inhibited progression of HCC possibly through regulating proliferation, stemness, and apoptosis.

Recently, Puerarin 6″‐O‐xyloside was characterized as a specific inhibitor of histone demethylation lysine‐specific demethylase 6B (KDM6B, also called jumonji domain‐containing protein 3 or JMJD3) with an IC50 value of 30.2 μmol/L and a Ki value of 7.5 μmol/L.^18^ KDMs play important roles in the epigenetic regulation of gene expression, especially in hypoxia and drug resistance. For example, KDM6A directly senses oxygen. KDM6A promotes H3K27 demethylation under hypoxia to block cellular differentiation.^19^ Hypoxia is the hallmark of solid tumors, and it was indicated that KDM6B was induced by HIF1A, the pivotal hypoxia‐inducible protein, in human and mouse.^20^ Overexpressed KDM6B promoted hepatoma cell migration, proliferation, and stemness, and inhibited apoptosis, thus promoting HCC carcinogenesis.^21^ KDM6B in clinical specimens of HCC was correlated inversely with patient survival, and this KDM6B overexpression induced EMT, stemness, and metastasis.^22^ Furthermore, KDM6B induced drug resistance in multiple tumors. Inhibition of KDM6B enhanced apoptotic response to PI3K/AKT inhibitor treatment in GDC‐0941‐resistant breast cancer cells.^23^ In addition, KDM6B was also involved in resistance of non‐solid tumors such as large B‐cell lymphoma.^24^ Consequently, inhibition of KDM6B showed promising effects in vivo in specific tumors like high‐risk neuroblastoma.^25^ So inhibition of KDM6B might be effective to HCC. Puerarin 6″‐O‐xyloside dose dependently inhibited proliferation and stemness, and promoted apoptosis in this study. These effects were possibly resulted from inhibited demethylation that was consistent with the effects of other KDMs.^21^ However, downstream of KDM6B was not tested at present, and to what extent Puerarin 6″‐O‐xyloside functioned through inhibiting KDM6B was not determined yet.

PI3K/AKT/mTOR signaling is an essential upstream of autophagy, drug resistance, proliferation, and stemness and important therapeutic target that dysregulated in more than 40% of HCC patients.^26^ However, PI3K inhibitors used as a monotherapy have shown limited clinical outcome, possibly as a consequence of resistance and poor tolerability.^27^ Co‐administration of PI3K/AKT/mTOR inhibitor with other targeted therapies and development of multi‐targeted chemicals have showed promising effects in vitro and in vivo.^28^, ^29^ Inhibition of PI3K or mTOR, or in combination is different. Inhibition of mTOR alone sometimes promoted drug resistance by PI3K activating feedback, and mTOR inhibition has been testified to be beneficial for the sensitivity to PI3K inhibitors. As a result, a series of 4‐acrylamido‐quinoline derivatives, as dual inhibitors of PI3K and mTOR, showed promising biological profiles.^30^ Puerarin 6″‐O‐xyloside decreased the relative expression of p‐PI3K, p‐AKT, and p‐mTOR and induced autophagy dose dependently, and PI3K inhibitor 3‐MA enhanced this effect. The effects of Puerarin 6″‐O‐xyloside on PI3K/AKT/mTOR signaling indicated that it could possibly target PI3K and mTOR at the same time. As expected, co‐administration of Puerarin 6″‐O‐xyloside and 3‐MA more significantly inhibited proliferation and stemness, and promoted apoptosis in HepG2 cells.

Very interestingly, other than 4‐acrylamido‐quinoline derivatives, Puerarin 6″‐O‐xyloside shared structural similarities with fused pyrimidine‐based hydroxamates, a series of PI3K/AKT/mTOR, and class I histone deacetylases dual inhibitors.^30^, ^31^ The fused pyrimidine‐based hydroxamates showed significant single agent oral efficacy in hypervascular liver cancer models. The similarities in structure and targets as well as similar effects provide new horizon for optimizing these compounds. On the other hand, multi‐targeted chemicals, such as Puerarin 6″‐O‐xyloside, may have side effects on normal tissues. For instance, activation of PI3K/AKT often exerts protective effects. The activation of the Lyn/PI3K/Akt pathways by a green barley extract exerted a significant reduction in dead cells when undergoing aggressive oxidative stress.^32^ The mechanism of action of Puerarin 6″‐O‐xyloside needs to be carefully explored.

## 5 ETHICAL APPROVAL STATEMENT

All the mice received human care and all experiments were done according to the guidelines of *the Animal Welfare Act and the Guide for Care and Use of Laboratory Animals from the National Institutes of Health*. The experimental protocols were approved by the Hunan Science and Technology Department (SYXK 2019‐0017) and in accordance with *the Principles of Human Experimental Technique* and with implications for replacement, refinement, or reduction (the 3Rs) principle.

## CONFLICT OF INTEREST

The authors declare no conflict of interest.

## CONFLICT OF INTEREST

The authors declare no conflict of interest.

## AUTHORSHIP STATEMENT

Hongbo Li and Long Li designed the research; Long Li, Jun‐Dong Liu, Guo‐Dong Gao, and Yu‐Wei Song performed the experiments; Jun‐Dong Liu and Kai Zhang collected the data; Yu‐Wei Song did the analysis; Hongbo Li drafted the manuscript; Hongbo Li revised the manuscript. All authors approved the final manuscript.

## Data Availability

All data are available upon request.
